The article "Research on the Relationship between Employee Mental Health and Enterprise Work Performance" was retracted in 2023. Reasons: signs of a paper mill; suspected computer-generated content; unreliable results or conclusions; concerns about the data.

# Research on the Relationship between Employee Mental Health and Enterprise Work Performance

**DOI:** 10.1155/2022/3008947

**Published:** 2022-02-27

**Authors:** Ningning Yan

**Affiliations:** School of Management and Economics, Jingdezhen Ceramic University, Jingdezhen 333403, China

## Abstract

Knowledge, capabilities, and quality can be used as three temperatures in employee value-added characteristics in corporate employee performance. They are closely coupled, and knowledge is the basis of ability and quality. The ability is to form and develop in the process of mastering knowledge. The quality is a potential ability. The quality itself is not the ability. Quality is a relatively stable quality and accomplishment formed by internalizing knowledge and skills acquired from the outside into people's body and mind through individual cognition and social practice on the basis of innate physiology and under the influence of acquired environment and psychology. Quality determines whether the employee's knowledge and ability can function correctly and effectively, and is the director of knowledge capabilities. According to the analysis and learning from scholars of literature employees' job performance evaluation, we constructed an employee performance evaluation index system of evaluation on the basis of value-based employees. In this system, there are three levels of evaluation indicators. The level indicators are as follows: knowledge of value-added indicators, the ability to add value, and quality index value. These indicators are consistent with the analysis of employee training objectives and psychological quality. In this study, for each level of each indicator we have specific labeling instructions, which is more convenient for the relevant calculations.

## 1. Introduction

As we all know, the high and low level of employee's starting point is very large, and the traditional evaluation neglects the difference in employee starting point. It adopts the same evaluation standard to evaluate obviously unfair, seriously damaging employee work. Enthusiasm: value-added employee evaluation is closely linked to employee's evaluation of employees, These indicators are consistent with the analysis of employee training objectives and psychological quality. Therefore, the health analysis is most different from traditional evaluation, and that is, it is very payable of employee's psychological starting point and is a dynamic evaluation [1].

The evaluation of mental health is a development range, pay attention to the psychological process, and prompt feedback. The main feature of this evaluation is to emphasize the authenticity and accuracy of employee development, and the evaluations and evaluation targets cooperate with each other to promote the future development of the evaluation. This evaluation method can improve the evaluation target and participate in the enthusiasm of psychological evaluation and the awareness of group [2]. It pays attention to the application of qualitative analysis and statistical methods, which not only attaches importance to evaluation results but also more importantly pays attention to full evaluation and comprehensive evaluation, emphasizing the quality of the work and also the process of development.

The value-added psychological evaluation requires the performance responsibility of enhancing the work of employees as marking the performance of the company and the employee, including developmental philosophy. According to the needs of psychological development, the United States has gradually formed a new psychological evaluation concept on the basis of reflecting traditional evaluation, and the development of mental health and the development of employee's career development and quality improvement. The main content of the value-added psychological evaluation is to collect the tests of employees in front and rear psychological knowledge, skills, quality, and after comparison, the knowledge, ability, and quality growth of employees during the work are analyzed. Then it makes a comprehensive evaluation of the psychological efficiency and work efficiency of the enterprise [3].

It uses the static evaluation method to perform longitudinal comparisons, and on the one hand, it is possible to accurately analyze the professionalism and work status of each employee and use dynamic developed eyes to see employees. On the other hand, it pays attention to the historical situation of a company and to the development potential and development trend of the company. Value-added psychological evaluation not only pays attention to the final psychological achievement of work but also emphasizes the development of employees, the development of employee work, and the development of corporate psychological benefits [4]. This can mobilize the enthusiasm, improve work, and improve the psychological process to provide more appropriate help and guidance.

First, through health evaluation, the development of employee work can be combined with employee evaluation and even enterprise evaluation and can enhance the objectivity of evaluation.

The famous American psychologist sanders and lavers proposed the employee of employees with high mental efficiency, and the employee's occupational value added very significant difference. The difference is high enough to have a decisive impact on the future occupation of the employee. This proves that the basic hypothesis of health evaluation is true. The difference in working conditions and concentration work at the time of participation of employees, that is, the changes in the development of employees, can be attributed to corporate psychology; the increase in employee development, that is, employee value-added, can be seen as a business, employee, or work. In this sense, the health evaluation is concerned with the development of employees. Whether as a means of employee evaluation, it is also a way to evaluate a business assessment, and its evaluation is more objective and fair. In addition, in the health evaluation, each employee is compared with the past career situation and the past career status, and highlights the objectivity of the evaluation.

In addition, in terms of evaluation methods, the analysis method for the evaluation of health is relatively complex and complete, in particular hierarchical analysis-fuzzy evaluation comprehensive analysis method for systematic analysis of “value-added” data obtained in the value-added evaluation process. Using this method, the health evaluation can exclude other interference factors that affect employees and corporate psychological effects; collect effective data such as employees' psychological foundation, intelligence level, working ability and cultural quality for objective evaluation [5].

## 2. Index Design of Enterprise Employee Work Performance Evaluation System

### 2.1. Selection of Evaluation System Index

The fundamental purpose of corporate employee's work performance assessment is to improve the quality of employees to achieve employee training targets.

#### 2.1.1. Employees' Knowledge Value-Added Indicators: Both Broad and Specialization

In the evaluation system, there are two indicators of value-added knowledge of two employees: extensive knowledge of special precision and knowledge. Knowledge training objectives and indicators are an important part of the work, which is one of the main advantage and disadvantage measures of the quality of staff development, primarily associated with employee growth mode learning system in its formation. One of the tasks of staff development mode is to give each employee a “unique knowledge structure in line with social needs and to adapt to personal characteristics.” Knowledge index: an important feature of the design is to promote a profound knowledge to promote staff development, emphasizing on the basis of knowledgeable staff specialization expertise [6]. Firstly, companies that develop extensive knowledge of employees in the learning system are mainly reflected in the more professional knowledge set. Numerous professional knowledge is the cornerstone of the enterprise, and the corporate culture is a broad characterization. Secondly, employees have extensive knowledge of design and are also reflected in the store's rich cultural resources.

Therefore, the so-called extensive expertise and knowledge of structural design not only have a broad base of knowledge but also have a solid professional knowledge and have the social, economic, and cultural development to match the knowledge system.

#### 2.1.2. Employee's Ability to Add Value Indicators: Theory and Practice

Ability comes from mastery of knowledge, and systematic and structured knowledge base is a necessary element. On the other hand, it is a better ability to create knowledge and knowledge acquisition premise activities. Therefore, knowledge of tradition, and innovation and training for capacity development are two important aspects of the mental health staff training. In the evaluation index system, three secondary indexes are set up in this study: cultivate employees' ability to acquire and use knowledge independently in each link of work; cultivate staff's creative thinking ability in scientific research activities; enhance employees' oral communication skills in various academic activities [3].

The so-called work independently acquires and applies knowledge; only refers to the teaching and guidance of enterprise employees are inspired employees to understand the knowledge of the process and figure out methods to acquire knowledge, learn independent thinking, logical deduction, and reasoning; also refers to work process and participation in various social activities; and fully mobilize employees to explore and research capabilities.

The so-called creative thinking ability refers to the creative consciousness and innovative spirit of thinking activities, nonconformist, singular, seeking change, manifested as creatively proposing problems and creatively solving problems.

The so-called verbal ability refers to the use of oral language to express their thoughts and feelings, to achieve the ability to communicate with other purposes. Oral language plays a more direct and more extensive role than the written language of communication. The development of modern society has put forward higher and higher requirements for people's oral expression ability.

#### 2.1.3. The Quality of Employee's Value-Added Indicators: Science, Culture, and Humanity

While ensuring that the trained employees have a solid knowledge structure and excellent professional talents, the enterprise employees also pay attention to cultivating employees with comprehensive quality to meet the needs of today's society. In the process of employee training, enterprise employees can participate in the edification of humanistic knowledge, humanistic environment, and scientific and technological practice, so as to make employees have a psychological improvement process and improve their cultural taste, humanistic quality, and scientific quality. Therefore, in the evaluation system, there are three value-added secondary indicators of the quality of employees: cultural taste, humanities, and scientific quality.

The so-called cultural taste refers to people's material and spiritual life of the product to a certain extent, and it must be built on a foundation of cultural training on the main parties; moreover, it is the result of the relative enrichment and richness of material and spiritual cultural life. Cultural taste mainly by the daily quality of life, aesthetic taste, and taste understands the value of art composed of three areas.

The so-called cultural literacy refers to the ability of the human sciences research, knowledge, and humanities reflected in human subjects, in the spirit of human-centered—the inherent human quality. The staff of the enterprise should have both scientific literacy and rich humanistic spirit; both professional knowledge and sound personality.

The so-called scientific literacy refers to the basic conditions of contemporary business students to participate in scientific activities in the social life. It includes scientific knowledge, scientific ideas, scientific methods, scientific spirit, and scientific problems. The comprehensive expression is the desire to pursue science, the attitude of respecting science, the behavior of exploring science, and the effect of innovating science.  Table 1 is the evaluation index system based on value-added employee mental health and work performance.

### 2.2. AHP—Fuzzy Comprehensive Evaluation Method

#### 2.2.1. AHP Hierarchy Analysis

*(1) Basic Method and Step of Level Analysis Method*. The main working principle of the hierarchical analysis is to make complex problems into different factors by decomposition and arranged in a hierarchical structure in accordance with different relationships. The importance of this method is obtained in accordance with the completion of the nature, and the total data judgment is used, and the total plan is set, and the research, design, and decision of the system can be completed by four procedures. The program is completed.

First, carry out the analysis of the relationship between the elements of the system to form a hierarchical structure.

Second, the variety of elements is compared in accordance with the formulation of the same level according to the formulation of the criteria; third, the result of obtaining a matrix comparison weight is calculated by the system.

Fourth, the sort of the weighting element is calculated by the system.

*(2) Establishment of the Hierarchical Structure*. The system structure model must be combed into a hierarchical, logical data model. In this structure, complex problems will not exist, and replaced is a decomposition element. At the same time, these elements are divided into several groups depending on the nature and are formed into different levels of data architectures. A variety of elements at the same level can be disposed of as a criterion to the next level element. Moreover, it is necessary to accept guidance from the previous level when the dominance is completed [7]. There are three levels.

One is the highest layer: on this level, there is only one, and its function is to complete the target setting and expectation of the problem, so there is another nameless target layer.

The second is the intermediate layer: the elements existing in this level are guidelines, which have hierarchical dominance, and there are other hierarchies in this level. These other levels are mainly general guidelines and submissions, so there are other names of the guidelines.

The third is the bottom layer: at this level, there is mainly decision-making plan, and the main work function is the development of the target program and strategic measures, so there is another name layer.

An important part of the hierarchical part of the order is hierarchical, which is formed by a dominant relationship formed by the upper and lower elements. However, the high level of high elements completes all elements of low levels and can also be administered by some elements. The composition of the hierarchical element of the order level directly affects the complexity of the problem, but also has an impact on the level decomposition of complex problems, but the hierarchical structure is not limited by complex problems. Generally speaking, elemental data existing in each decomposition are less than or equal, mainly because if the number of elements is too large, the inaccuracies of two judges will be caused. The reasonable extent of the decomposition hierarchy directly determines the advantages and disadvantages of complex problems, but it is important to establish a multi-element hierarchical structure and decision-makers have an important relationship with complex issues.

*(3) Construction of Two Comparison Judgment Matrices*. In the hand-order hierarchy matrix, assume that the previous element *C* is set to the standard, and the C criterion corresponding to the next element of *u*_2_,…, and *u*_*n*_ is the weight. There are generally two cases.

First, if the importance of *u*1, *u*2,…, *u*_*n*_ to *C* can be quantified, then the weight can be determined.

Second, if the problem is more complicated and *u*_1_, *u*_2_,…, *u*_*n*_ is unable to quantify the importance of *C*, which can only be a qualitative analysis, then the weight can be completed by two comparison methods. The main steps are as follows: relative to C criterion, which element ui and uj is suitable for, and which program is suitable for, the numerical comparison of important programs is generally completed according to the scale of one to nine.  Table 2 shows the meaning of the scale of one to nine.

For criterion C, the importance of the construction of *n* elements is obtained through the comparison of pairwise matrices.

(1) $$\begin{array}{c} A={\left(a_{ij}\right)}_{n\times n}. \end{array}$$

Here, *a*_*ij*_ represents the proportional scale of elements *u*_*i*_ and *u*_*j*_ relative to the important setting of C criterion. The properties of matrix A are determined as follows: *a*_*ij*_ > 0, *a*_*ji*_=1/*a*_*ij*_, and *a*_*ii*_=1.

Through the judgment of matrix properties, it is concluded that the judgment of *n* elements in the matrix can be completed using *n* (*n* − 1)/2 elements in the triangle above or below the matrix. That is, as long as there are *n* (*n*− 1)/2 in the matrix, the pairwise comparison can be completed.

If matrix A can satisfy all elements *a*_*ij*_•*a*_*jk*_=*a*_*ik*_, then a is the consistency matrix.

Not all judgment matrices can meet the conditions, but they can meet the conditions of complex problems only in special cases.

*(4) Calculation of Element Relative Weight under Single Criterion and Consistency Test of Judgment Matrix*. It is known that the *n* elements *u*1, *u*2,…, *u*_*n*_ determine the a matrix for the C criterion, and the absolute weight *ω*_1_, *ω*_2_,…, *ω*_*n*_ of *u*1, *u*2,…, *u*_*n*_ is calculated for the C criterion, which can be expressed as *W*=(*ω*_1_, *ω*_2_,…,*ω*_*n*_)^*T*^.

First is the method of calculating the weight.

(a) Law. After the *n* row vectors of matrix A are judged and calculated, the value obtained is the weight vector, as shown as follows:
  (2) $$\begin{array}{c} \omega_{i}=\sum_{j=1}^{n}\frac{a_{ij}}{n\sum_{k=1}^{n}a_{kj}}\;i=1,2,\ldots ,n. \end{array}$$
The main steps are as follows: the normalization of element a is completed and added according to the normalized hierarchy. The added vector is divided by *n* to obtain the weight vector.
There are other methods, such as column and normalization:
  (3) $$\begin{array}{c} \omega_{i}=\frac{\sum_{j=1}^{n}a_{ij}}{n\sum_{k=1}^{n}\sum_{j=1}^{n}a_{ij}}\;i=1,2,\ldots ,n. \end{array}$$
The root method is the geometric average method we usually use. After the vector average of *a* is completed, the value obtained through normalization calculation is the weight vector. The calculation formula is as follows:
  (4) $$\begin{array}{c} \omega_{1}=\frac{{\left(\prod_{j=1}^{n}a_{ij}\right)}^{1/n}}{\sum_{k=1}^{n}{\prod_{j=1}^{n}a_{kj}}^{1/n}}\;i=1,2,\ldots ,n. \end{array}$$
The main steps are as follows: the vector multiplication of element *a* is completed; after multiplication, the *n*th power is found; after the calculated vector is normalized, the weight vector is obtained.
The characteristic root method is the commonly used EM method. The main function is to complete the characteristic solution of matrix A.
  (5) $$\begin{array}{c} AW=\lambda_{\max}W. \end{array}$$
Here, *λ*_max_ is the largest eigenvalue of *a*, and *W* represents the corresponding vector. The obtained result *w* obtains the weight vector after normalization calculation.
(b) Logarithmic least squares. Through the comparison of the two methods, the weight vector is determined as *W*=(*ω*_1_, *ω*_2_,…,*ω*_*n*_)^*T*^, and the obtained square residual and the minimum values are as follows:
  (6) $$\begin{array}{c} \sum_{1\leq i\leq j\leq n}1ga_{ij}-1g\left(\frac{\omega_{i}}{\omega_{j}}\right). \end{array}$$
(c) Least-squares method. The weight vector *W*=(*ω*_1_, *ω*_2_,…,*ω*_*n*_)^*T*^ is set, and the square of the residual and ∑_1≤*i*≤*j*≤*n*_[1*ga*_*ij*_ − 1*g*(*ω*_*i*_/*ω*_*j*_)]^2^ are determined as the minimum values.

Second is the consistency test.

The weight vector can be calculated only through the consistency test. In the matrix, it is not particularly emphasized whether *a*_*ij*_•*a*_*jk*_=*a*_*ik*_ is equal, but it can meet the consistency. If there are fuzzy data, it violates the objectivity of judgment, resulting in matrix decision-making error. For the above weight calculation method, because the deviation of the matrix reduces the reliability performance, the matrix inspection should be further completed. The main procedures are as follows:

(a) The consistency index (C.I.) is obtained as follows:
  (7) $$\begin{array}{c} C.I.=\frac{\lambda_{\max}-n}{n-1}. \end{array}$$
(b) The corresponding average value (R.I.) is found.
Table 3 is the average random consistency index (R.I.).
(c) The data scale (C.R.) is calculated as follows:
  (8) $$\begin{array}{c} C.R.=\frac{C.I.}{R.I.}. \end{array}$$

When C.R.< 0.1, the matrix that meets the consistency requirements is determined; when C.R.≥ 0.1, the matrix value must be modified.

The consistency can be determined by calculating the maximum eigenvalue *λ*_max_ of the matrix. Other methods can also be used. The main formulas are as follows:

(9) $$\begin{array}{c} \lambda_{\max}=\sum_{i=1}^{n}\frac{{\left(AW\right)}_{i}}{n\omega_{i}},\\ =\frac{1}{n}\sum_{i=1}^{n}\frac{\sum_{j=1}^{n}a_{ij}\omega_{i}}{\omega_{i}}. \end{array}$$

The total sorting weights of elements in different levels and total target levels are obtained. The weight vector of the element in the previous level can be obtained. To get all the elements, the sorting weight of the next level objectives, that is, the total sorting weight, must be calculated to complete the scheme comparison.

If *W*^(*k* − 1)^=(*ω*_1_^(*k* − 1)^, *ω*_2_^(*k* − 1)^,…,*ω*_*k*−1_^(*k* − 1)^)^*T*^ represents *n*_*k*−1_elements and sorting weight vector in *k* − 1 level and *P*_*j*_^(*k*)^=(*p*_1*j*_^(*k*)^, *p*_2*j*_^(*k*)^,…,*p*_*n*_*k*_,*j*_^(*k*)^)^*T*^ represents the weight vector of *n*_k_ elements in *k* level and *j* elements in *k* − 1 level, the element weight dominated by *j* element is 0. *P*^(*k*)^=(*p*_1*j*_^(*k*)^, *p*_2*j*_^(*k*)^,…,*p*_*n*_*k*_,*j*_^(*k*)^)^*T*^ stands for *n*_*k*_ × *n*_*k*−1_ matrix ladder, which represents the arrangement order of elements *k* − 1 in layer *k*, and it is concluded that the total arrangement of elements in layer *k* is *W*^(*k*)^:

(10) $$\begin{array}{c} W^{\left(k\right)}={\left(\omega_{1}^{\left(k\right)},\omega_{2}^{\left(k\right)},\ldots ,\omega_{n_{k}}^{\left(k\right)}\right)}^{T}=P^{\left(k\right)}•W^{\left(k-1\right)},\\ \text{or}\\ \omega_{j}^{\left(k\right)}=\sum_{j=1}^{n_{k-1}}p_{ij}^{\left(k\right)}\omega_{j}^{\left(k-1\right)}\;i=1,2,\ldots ,n_{-}. \end{array}$$

The general formula is *W*^(*k*)^=*P*^(*k*)^*P*^(*k* − 1)^ … *W*^(2)^, where (*W*^2^) represents the ranking of the total elements of the upper layer.

If the consistency test from the previous level to the next level is to be completed, it must be calculated that the element *J* in layer *k* − 1 represents the consistency index C.I. *j*(*k*), the consistency value of any sample is R.I. *j*(*k*), and the similarity ratio C.R. *j* (*k*) (where *j* = 1, 2,…, *n*_*k*−1_), and all the indexes of layer *k* are as follows:

(11) $$\begin{array}{c} C.I.^{\left(k\right)}=\left(C.I._{1}^{\left(k\right)},\cdots ,C.I._{n_{k-1}}^{\left(k\right)}\right)•W^{\left(k-1\right)},\\ R.I.^{\left(k\right)}=\left(R.I_{-1}^{\left(k\right)},\cdots ,R.I_{\cdot n_{k-1}}^{\left(k\right)}\right)•W^{\left(k-1\right)}. \end{array}$$

When C.R. (*k*)<0.1, it can be determined whether the calculation results in different levels and the weight in layer *k* include the consistency and satisfaction of data.

#### 2.2.2. Fuzzy Comprehensive Evaluation Method

Fuzzy comprehensive evaluation method is a method and tool to effectively analyse and judge the fuzzy system according to the basic principles of fuzzy mathematics. This method is based on the relationship between qualitative and quantitative, unifies the accurate and imprecise ideas with the processing method of fuzzy mathematics, and has unique advantages in the complex system evaluation, which is difficult to express in detail. The fuzzy comprehensive evaluation method includes single-level fuzzy comprehensive evaluation model and multilevel fuzzy comprehensive evaluation model.

In two given sets *U* = {*u*1, *u*2,…, *um*} and *V* = {*v*1, *v*2,…, *vn*}, set *U* represents all evaluation elements and *V* represents the evaluation level set.

Let *ui* be the *i*th evaluation factor, and then, the single factor evaluation result is *Ri* = [*r*_*i1*_, *r*_*i2*_,…, *r*_*in*_]; thus, the decision matrix of *m* evaluation factors is *R*:

(12) $$\begin{array}{c} R=\left[\begin{array}{c} R_{1}\\ R_{2}\\ \vdots \\ R_{n} \end{array}\right]\\ =\left[\begin{array}{cccc} r_{11} & r_{12} & \cdots & r_{13}\\ r_{21} & r_{22} & \cdots & r_{23}\\ \vdots & \vdots & \ddots & \vdots \\ r_{m1} & r_{m2} & \cdots & r_{mn} \end{array}\right]. \end{array}$$

Here, *R* is a fuzzy relation representation of *U* ⟶ *V*. If the weight of the evaluation elements is analyzed and its set a is obtained, it is obvious that this set is *A*=[*a*_1_, *a*_2_,…, *a*_*m*_] fuzzy subset of *U*, and at the same time, 0 ≤ *a*_*i*_ ≤ 1, ∑_*i*=1_^*m*^*a*_*i*_=1. According to the operation principle of fuzzy transformation, a fuzzy subset of its corresponding relationship set *V* can be obtained, that is, the evaluation result *B*=*A* × *R*=[*b*_1_, *b*_2_,…, *b*_*n*_].

*(1) Multilevel Fuzzy Comprehensive Evaluation Model*. The single-level fuzzy comprehensive evaluation model is simple and easy to use, but it is insufficient to evaluate large-scale complex systems, because there are many elements in these systems, and these elements are interrelated and affect each other. Therefore, we can classify the set of evaluation elements, judge each type of elements, and then judge between classes. This is the principle of multilevel fuzzy comprehensive evaluation model, and its theoretical basis is still consistent with the single-level fuzzy comprehensive evaluation model. The operation steps of the multilevel fuzzy comprehensive evaluation model are as follows:

Firstly, the evaluation factor *U* is established. According to a classification method, *U* is divided into several subsets, and the following conditions are met:

(13) $$\begin{array}{c} \left\{\begin{array}{c} \sum_{i=1}^{m}Ui=U,\\ U_{i}\cap U_{j}=\Phi \left(i\neq j\right). \end{array}\right) \end{array}$$

From the above formula, the set of evaluation elements at the next level can be obtained; that is, *U* = {*U*1, *U*2,…, *Um*}. In this equation, *Ui* = {*Uik*} (*i* = 1, 2,…, *m*; *k* = 1, 2,…, *nk*) indicates that the subset UI contains *nk* evaluation factors.

Secondly, according to the principle of single-level fuzzy comprehensive evaluation model, the evaluation elements in *Ui* are analyzed. If the weight is *Ai* and the decision matrix is *Ri*, the comprehensive evaluation result *Bi* of *Ui* is obtained:

(14) $$\begin{array}{c} B_{i}=A_{i}\times R_{i}=\left[b_{i1},b_{i2},\ldots ,b_{in}\right]. \end{array}$$

Finally, several evaluation factor subsets of *U* set are comprehensively evaluated, and the decision matrix *R* is expressed as follows:

(15) $$\begin{array}{c} R=\left[\begin{array}{c} B_{1}\\ B_{2}\\ \vdots \\ B_{n} \end{array}\right]\\ =\left[\begin{array}{cccc} b_{11} & b_{12} & \cdots & b_{13}\\ b_{21} & b_{22} & \cdots & b_{23}\\ \vdots & \vdots & \ddots & \vdots \\ b_{m1} & b_{m2} & \cdots & b_{mn} \end{array}\right]. \end{array}$$

If the weight is *A*, the comprehensive evaluation result can be obtained, and *B*^*∗*^ is expressed as follows: *B*^*∗*^=*A* × *R*. This result *B*^*∗*^ is the final judgment result. Of course, if there are many elements in *U*, it can be divided many times according to the above methods and a multilevel fuzzy comprehensive evaluation model can be established, which can not only overcome the problems of different levels of elements, but also avoid the problem that it is difficult to determine the weight.

#### 2.2.3. Analysis Steps of AHP Fuzzy Comprehensive Evaluation

1. Questionnaire survey, through expert survey method, concentrated opinion method, or Delphi method to obtain data. After the construction of the evaluation system, the relevant evaluation needs two types of data support: firstly, the index weight is determined, and the mutual weight of different levels of indicators is judged by inviting experts to score the indicators; secondly, experts in relevant fields should score the lowest indicators according to the fuzziness. In the process of obtaining these two kinds of data, it should be noted that well-known experts or authoritative experts in relevant fields must be selected to improve the reliability of weight and the validity of data; at the same time, in the process of questionnaire design, the questionnaire should be modified repeatedly through pre-survey, and finally, a scientific, reasonable, hierarchical, and effective questionnaire should be designed, and the effective recovery rate of the questionnaire should be guaranteed in the process of data collection.
2. Determining the weight of indicators
3. In the analytic hierarchy process, the determination of weight should follow the principle of top-down. Firstly, the weight vector of the primary index (criterion layer) is determined, and the element of the weight vector is actually the fuzzy membership degree. In the AHP fuzzy comprehensive evaluation, we can determine the importance level of the index through the AHP analysis method, so as to obtain the relevant weight and normalize it, that is, to make ∑_*i*=1_^*p*^*a*_*i*_=1. Secondly, the weights of the domain layer and the index layer can also be determined. Finally, experts are invited to score the relative importance of the last level index to the target layer.
4. Using fuzzy comprehensive evaluation method to evaluate the level of competitiveness.

Firstly, the factor set of the evaluation object is determined, that is, to establish a reasonable set of evaluation factors according to the evaluation index system set in this study.

Secondly, the rating set of comments is determined. The evaluation grade set reflects the different states of evaluation indicators, which can be evaluated and graded by experts.

(16) $$\begin{array}{c} \left[\begin{array}{cccc} r_{11} & r_{12} & \cdots & r_{1\sigma }\\ \cdots & \; & \; & \;\\ r_{\sigma 1} & r_{\sigma 2} & \cdots & \; \end{array}\right]. \end{array}$$

Thirdly, the fuzzy relation matrix *R* is established.

Fourthly, the fuzzy comprehensive evaluation result vector is synthesized. The set *A* is synthesized with the evaluated *R* to obtain the result vector *B*.

Fifthly, the result vector of fuzzy comprehensive evaluation is analyzed. The evaluated indexes according to the maximum membership degree or average weighted membership degree are ranked.

## 3. Empirical Research

Firstly, the evaluation object is determined. The evaluation objects of this study are 170 representative enterprise employees' job performance.

Secondly, the evaluation factor set is set. The evaluation factor set is *u* = {*u*1, *u*2, *u*3,…, *u*23} = {diversity of contents, flexibility of working methods, richness of working resources, depth of knowledge, firmness of knowledge, mastery of practical operation knowledge, independent thinking, logical derivation and demonstration, exploration ability, research ability, creative problem-raising, creative problem-solving, expressing their thoughts and emotions, enhancing communication, daily life quality and art Artistic aesthetic taste, value understanding taste, humanistic spirit, sound personality, respect and work scientific beliefs and attitudes, explore scientific behavior, and innovate scientific results}.

Thirdly, the comment set is determined. According to the actual needs of evaluation and decision-making, the evaluation grade standard is divided into five grades: “good,” “good,” “general,” “poor,” and “poor.” *V* = {*v*1, *v*2, *v*3, *v*4, *v*5} = {good 5, good 4, average 3, poor 2, poor 1}.

Finally, due to the need for matrix operation in the fuzzy comprehensive evaluation, DPS14.1 software is used to calculate and get the final result. The English name of DPS is data processing system, which is abbreviated as DPS. DPS platform is a general multifunctional mathematical statistics and mathematical model processing software system designed and developed by the author. It integrates the functions of numerical calculation, statistical analysis, model simulation, and line drawing and tabulation. Therefore, DPS is mainly used as a data processing and analysis tool for the majority of users.

At the same time, according to the actual situation of employees' work performance evaluation, we set the comprehensive competitiveness evaluation score of more than 3.5 as the good level, 3.3–3.5 as the medium and upper level, and below 3.3 as the general level.

After DPS software calculation, we can get the comprehensive evaluation results of secondary indicators as shown in Table 4, the comprehensive evaluation results of primary indicators as shown in Table 5, and the overall evaluation results of comprehensive competitiveness as shown in Table 6.

## 4. Analysis of Evaluation Results

### 4.1. Analysis of Evaluation Results of Secondary Index and Primary Index

#### 4.1.1. Analysis of Secondary Index Evaluation Results

As shown in Table 4, among the average secondary indicators of 17 enterprises, the indicators with a score of more than 3.5 include professional knowledge accuracy (3.50829), creative thinking ability (3.50259), and scientific quality (3.90790). Among them, the highest score is scientific quality. The high score of scientific quality index fully reflects the current practical needs of enterprise employees for employees' work. Only enterprise employees who master basic scientific methods establish scientific ideas and advocate scientific spirit can have a foothold in the society, which also requires enterprise employees to pay more attention to the cultivation of employees' scientific quality in their work. On the other hand, the score of the ability index of acquiring and applying knowledge is only 3.21976, indicating that the employees of 17 enterprises still lack knowledge appreciation. In particular, there are serious deficiencies in guiding employees how to work and apply unfamiliar knowledge. Some employees are satisfied with reading in class and inculcating book knowledge.

#### 4.1.2. Analysis of Primary Index Evaluation Results

As shown in Table 5, the average scores of the three first-level indicators of knowledge value-added, ability value-added, and quality value-added in 17 enterprises are 3.407832, 3.267929, and 3.522625, respectively.

### 4.2. Analysis of Comprehensive Evaluation Results

As shown in Table 6, the average of the final evaluation results of employees' work performance in 17 enterprises is 3.368436. According to the principle of maximum membership, the evaluation of employees' work performance in these enterprises is above the national average level and close to a better level. Among them, 5 enterprises are at a good level, accounting for 29.4%; seven enterprises are at the upper-middle level, accounting for 41.2%; and five enterprises are at the general level, accounting for 29.4%. However, in reality, there is still a big gap between the results of job performance evaluation of employees in these enterprises and first-class enterprises.

## 5. Conclusions

Although the quality of employees in China's enterprises is constantly improving, and the working methods, working levels, and working means are constantly improving, how to improve the acquisition and practical application ability of employees' theoretical and practical knowledge is still insufficient. This is also the fundamental reason why it is difficult for some large employees to find employment after graduation, which has become a bottleneck in the current enterprise reform and development. From this score, the quality appreciation score is relatively high, which fully shows that under the call of the current quality psychology, all enterprises and competent departments pay attention to it, and the scientific spirit and humanistic quality of employees have been significantly improved. However, the scores of knowledge value-added and ability value-added are not satisfactory, which is related to the lack of in-depth reform of employees' work in Chinese enterprises. We can find key indicators to improve. At the same time, we find that the evaluation value of knowledge specificity is higher than that of knowledge breadth; the evaluation value of creative thinking ability is greater than oral expression ability, and oral expression ability is greater than the ability to acquire and apply knowledge; scientific quality is greater than cultural quality, and cultural quality is greater than humanistic quality. These results fully reflect the achievements of the current enterprise work reform in China. In general, according to the established evaluation index system, this study evaluates and analyzes the job performance of some typical enterprise employees in Beijing, Zhejiang, Liaoning, Henan, Hunan, Hubei, and Jiangxi. The evaluation results basically reflect the current situation of employee performance in these enterprises, which also fully shows the scientificity and objectivity of the evaluation index system constructed by this study.

## Figures and Tables

**Table 1:** Evaluation index system based on value-added employee mental health and work performance.

Target layer	Criterion layer	Field layer	Indicator layer
Work performance evaluation index system A	First-class indicator (B)	Secondary indicators (C)	Three-level indicator (D)
	Knowledge value B1	Knowledge broad C1	Content diversity D1
			Flexibility of working mode D2
			Work resource-rich D3
		Knowledge specialization C2	Depth of knowledge D4
			Solidity D5
			Mastering the actual operation knowledge D6
	Ability value B2	Get and use the ability to use knowledge C3	Independent thinking D7
			Logical derivation and argumentation D8
			Exploration capability D9
			Research capacity D10
		Create thinking C4	Creatively propose problems D11
			Creatively solve problems D12
		Verbal expression C5	Express your own ideas D13
			Express your emotions D14
			Enhance communication D15
	Quality value B3	Cultural taste C6	Daily life taste D16
			Art aesthetic taste D17
			Value understanding D18
		Humanism C7	Humanistic spirit D19
			Healthy personality D20
		Scientific quality C8	Respect scientific beliefs and attitude D21
			Explore scientific behavior D22
			Effectiveness of innovative science D23

**Table 2:** Scale and meaning.

Scale	Meaning
1	Represents the comparison of two elements, and the results include the same importance
3	Represents the comparison of two elements, and the result is that the former is more important
5	Represents the comparison of two elements, and the result is that the former is obviously important
7	Represents the comparison of two elements, and the result is that the latter is very important
9	Represents the comparison of two elements, and the result is that the latter is particularly important
2, 4, 6, 8	Represents the intermediate value of the above adjacent judgment
Reciprocal	If the ratio of the importance of elements *i*and *j* is *a*_*ij*_, then result of the importance of elements *j* and *i* is *a*_*ji*_=1/*a*_*ij*_

**Table 3:** Average random consistency index (R.I.) [8].

Matrix order	1	2	3	4	5	6	7	8
R.L	0	0	0.52	0.89	1.12	1.26	1.36	1.41
Matrix order	9	10	11	12	13	14	15	
R.L.	1.46	1.49	1.52	1.54	1.56	1.58	1.59	

**Table 4:** Comprehensive evaluation results of secondary indicators.

Enterprise	Extensive knowledge	Knowledge specialization accuracy	Ability to acquire and apply knowledge	Creative thinking ability	Oral expression ability	Cultural taste	Humanistic quality	Scientific quality
1	3.12287	3.98812	3.18281	3.3096	3.30305	3.229499	3.300496	4.396959
2	2.98837	3.502039	3.403092	2.89381	2.50092	3.129925	2.308912	4.120303
3	3.878391	3.76848	3.763638	3.12883	3.9494	3.78829	2.7838	4.20939
4	3.67474	3.48929	3.49995	3.102031	2.903936	3.794746	2.598841	3.787743
5	3.99842	2.988488	2.13321	3.9198	3.34818	3.12976	3.184881	4.16603
6	2.7319	3.14681	3.44789	3.26512	3.94699	3.94876	3.47211	3.93503
7	3.944905	4.32319	3.04875	4.2	3.0595	3.5485	3.44321	3.43355
8	4.4345	3.14092	2.439394	4.85881	3.49412	4.1	3.99932	3.11532
9	3.45763	4.25	3.4	3.31549	3.143572	3.132	3.44341	3.976514
10	3.100495	3.5	3.14379	3.38	3.46	3.981232	4.3	4.1345
11	3.94492	3.04049	2.99487	2.94985	3.343494	3.12923	4.88743	3.34945
12	2.99848	2.98472	3.243344	3.232312	3.232696	3.132444	3.43216	3.984311
13	3.34	3.43458	3.343332	3.35462	3.346885	3.434562	3.766282	3.498717
14	2.97748	3.194802	3.409381	3.348412	3.134559	3.23919	3.328181	3.874211
15	3.467103	3.929946	3.440949	4.39991	4.13844	3.123321	3.39191	4.123461
16	3.182766	3.192884	3.542618	3.397171	3.39299	3.821021	3.29102	4.198828
17	3.39821	3.766111	3.298812	3.488213	3.119391	3.7662112	3.1929392	4.12993
Mean value	3.44948	3.50829	3.21976	3.50259	3.34224	3.4958	3.41911	3.90790
Sort	2	1	3	1	2	2	3	1

**Table 5:** Comprehensive evaluation results of primary indicators.

Enterprise	Knowledge increment	Capability increment	Quality appreciation
1	3.49191	3.1700211	3.6162777
2	3.01192	2.8818287	3.1782998
3	3.69911	3.528819	3.5939884
4	3.58201	3.099291	3.328
5	3.37835	3.0625123	3.4000192
6	2.82821	3.388882	3.677372
7	4.0993	3.3293911	3.4885892
8	3.71823	3.41992912	3.3784889
9	3.78831	3.2300192	3.399492
10	3.257191	3.333948	4.001992
11	3.419982	3.000192	3.6747292
12	2.970112	3.12938499	3.4938881
13	3.3873	3.23887477	3.4775821
14	3.000012	3.21992923	3.3766466
15	3.655571	3.8877747	3.444883
16	3.156714	3.4000102	3.7666251
17	3.488919	3.233994	3.5877473
Average value	3.407832	3.267929	3.522625
Evaluation ranking	2	3	1

**Table 6:** Comprehensive evaluation results of employees' work performance.

Reorder sequence number	Comprehensive evaluation score	Ranking of evaluation by level
1	3.6019293	Relatively good
2	3.5593931	Relatively good
3	3.529192	Relatively good
4	3.52299	Relatively good
5	3.500787	Relatively good
6	3.4288371	Above average
7	3.401993	Above average
8	3.366176	Above average
9	3.3301	Above average
10	3.32839	Above average
11	3.3192911	Above average
12	3.310003	Above average
13	3.239	Ordinary
14	3.2388478	Ordinary
15	3.2199303	Ordinary
16	3.1892901	Ordinary
17	3.177263	Ordinary
Average value	3.368436	

## Data Availability

The simulation experimental data used to support the findings of this study are available from the corresponding author upon request.

## References

[1] Lieberman A., Pointer Mace D. H. (2008). Teacher learning: the key to educational reform. *Journal of Teacher Education*.

[2] Bartlett S. (2000). The development of teacher appraisal: a recent history. *British Journal of Educational Studies*.

[3] Weistroffer H. R., Spinelli M. A., Canavos G. C., Fuhs F. P. (2001). A merit pay allocation model for college faculty based on performance quality and quantity. *Economics of Education Review*.

[4] De Witte K., Rogge N. (2011). Accounting for exogenous influences in performance evaluations of teachers. *Economics of Education Review*.

[5] Borko H. (2004). Professional development and teacher learning: mapping the terrain. *Educational Researcher*.

[6] Allan O. (2004). Lessons learned about standards-based teacher evaluation systems. *Peabody Journal of Education*.

[7] Brennan J., Shah T. (2000). Quality assessment and institutional change: experiences from 14 counties. *Higher Education*.

[8] Zeng J.-h. (2012). Products selection modeling of medicine manufacturing industry development in Beibuwan economical zone. *International Journal of Wireless and Microwave Technologies*.

